This article has been retracted.

# Novel Mechanism of Inhibition of Dendritic Cells Maturation by Mesenchymal Stem Cells via Interleukin-10 and the JAK1/STAT3 Signaling Pathway

**DOI:** 10.1371/journal.pone.0055487

**Published:** 2013-01-30

**Authors:** Wen-hua Liu, Jing-jin Liu, Jian Wu, Lu-lu Zhang, Fang Liu, Li Yin, Mao-mao Zhang, Bo Yu

**Affiliations:** 1 Intensive Care Unit (ICU) Department, Second Affiliated Hospital of Harbin Medical University, Harbin, Province Heilongjiang, China; 2 Cardiology Department, Second Affiliated Hospital of Harbin Medical University, Harbin, Province Heilongjiang, China; Georgia Health Sciences University, United States of America

## Abstract

Mesenchymal stem cells (MSCs) can suppress dendritic cells (DCs) maturation and function, mediated by soluble factors, such as indoleamine 2,3-dioxygenase (IDO), prostaglandin E_2_ (PGE_2_), and nitric oxide (NO). Interleukin-10 (IL-10) is a common immunosuppressive cytokine, and the downstream signaling of the JAK-STAT pathway has been shown to be involved with DCs differentiation and maturation in the context of cancer. Whether IL-10 and/or the JAK-STAT pathway play a role in the inhibitory effect of MSCs on DCs maturation remains controversial. In our study, we cultured MSCs and DCs derived from rat bone marrow under different culturing conditions. Using Transwell plates, we detected by ELISA that the level of IL-10 significantly increased in the supernatants of MSC-DC co-cultures at 48 hours. The cell immunofluorescence assay suggested that the MSCs secreted more IL-10 than the DCs in the co-cultures. Adding exogenous IL-10 to the DCs monoculture or MSC-DC co-cultures stimulated IL-10 and led to a decrease in IL-12, and lower expression of the DCs surface markers CD80, CD86, OX62, MHC-II and CD11b/c. Supplementing the culture with an IL-10 neutralizing antibody (IL-10NA) showed precisely the opposite effect of adding IL-10. Moreover, we demonstrated that the JAK-STAT signaling pathway is involved in inhibiting DCs maturation. Both JAK1 and STAT3 expression and IL-10 secretion decreased markedly after adding a JAK inhibitor (AG490) to the co-culture plate. We propose that there is an IL-10 positive feedback loop, which may explain our observations of elevated IL-10 and enhanced JAK1 and STAT3 expression. Overall, we demonstrated that MSCs inhibit the maturation of DCs through the stimulation of IL-10 secretion, and by activating the JAK1 and STAT3 signaling pathway.

## Introduction

Mesenchymal stem cells (MSCs) are multipotent cells capable of differentiating into various lineages, including adipogenic, osteogenic, and chondrogenic [1]. MSCs are characterized by their expression of surface markers, such as CD29, CD90, and CD44, and the absence of the hematopoietic lineage markers CD34 and CD45 [2]–[4]. MSCs have unique characteristics, such as the previously reported low immunogenicity and immunoregulatory properties [5]–[9]. Recently, MSCs gained attention because of their immunosuppressive abilities against T cells [5], DCs [6]–[8], B cells [9], and natural killer (NK) cells [10]. Thus, MSCs are currently being used to reduce immunological rejection and prolong graft survival. Because dendritic cells (DCs) are the most potent antigen-presenting cells (APCs), they play a pivotal role in initiating immune response. Thus, it is important to study the mechanism(s) involved in the activity of the MSCs and the maturation of DCs. A few studies have demonstrated that IL-6, prostaglandin E2 (PGE2) and indoleamine-2,3-dioxygenase (IDO) may be implicated in MSCs-mediated inhibition of DCs function. Djouad *et al.* [11] observed that MSCs secrete higher levels of IL-6 which may be involved in reversing the maturation of DCs into a less mature phenotype, and in the partial inhibition of bone marrow progenitor differentiation into DCs. Chen *et al.* [12] demonstrated that blocking PGE2 synthesis in MSCs could revert most of the inhibitory effects on differentiation and function of DCs. In short, MSCs disrupt the transition of DCs from immature to mature states by secreting inhibitory soluble factors.

It is known that DCs play a key role in the initiation of primary immune responses and the induction of tolerance [13]. Normally, the life of DCs can be divided into two major phases [14] – an immature stage, and a mature stage [13], [15] that is associated with a high expression of molecules involved in antigen presentation (i.e., CD80, CD86, OX62, MHC-II, and CD11b/c). DCs maturation is a prerequisite for induction of immunogenic T cell responses. Recent studies have focused on the influence of bone marrow MSCs on the activity of DCs *via* specific signaling pathways [16], [17]. Therefore, we may conclude that MSCs modulate the differentiation, maturation, and function of DCs *via* the secretion of cytokines and /or activation of defined signaling pathways.

IL-10 is a potent immunosuppressive cytokine, produced primarily by Th2 cells, macrophages, and activated B cells [18].This cytokine has a wide range of biological activities, including immunosuppressive, anti-inflammatory and immunomodulatory properties, which regulate a variety of immune cell differentiation and proliferation events [19]. Corinti *et al.* [20] found that immature monocyte-derived DCs released sizeable amounts of IL-10. After stimulation with LPS, mDCs secreted high levels of IL-10 [21], which is known to inhibit DCs maturation and function. Thus, inhibiting the ability of DCs to produce IL-12, which is essential for driving Th1 cell differentiation. IL-10 can also down-regulate the major histocompatibility complex I (MHC-I) and growth and differentiation of B cells, T cells, DCs and other cells involved in inflammatory responses. Kim *et al*. [22] concluded that interleukin (IL)-10, induced by CD11b (+) cells and IL-10-activated regulatory T cells, play a role in the immune modulation of mesenchymal stem cells in rat islet allografts.

We herein formulate, and test, the hypothesis that MSCs may express IL-10 to influence the activity and maturation of DCs through a similar mechanism as regulatory T cells. Furthermore, we also propose a mechanism of action of IL-10-mediated inhibition of DCs that involves MSCs. Conzelmann *et al*. [23] reported that the JAK/STAT signaling pathway is strictly complementary for the induction of a pro-inflammatory cytokine profile in human antigen-presenting cells (APCs). We postulate that the downstream signaling pathway of JAK-STAT may be implicated in this specific inhibitory effect.

The JAK-STAT signaling pathway is one of the most important signal transduction cascades and is essential for the regulation of cytokine receptor signaling. When combined, the IL-10 and the IL-10 receptor activate the JAK1-STAT3 pathway [24]. Several studies [25], [26] have shown that the members of the STAT family, and more specifically STAT3, could be responsible for abnormal DCs differentiation and function in cancer. Hirata *et al.* [26] examined the role of JAKs in the regulation of inflammatory versus anti-inflammatory cytokine balance in murine conventional DCs. Blocking the JAK pathway by JAK inhibitor I (JAKi) resulted in significant inhibition of IL-10 production by DCs. JAKi completely blocked TLR-mediated STATs activation. In summary, these studies [24]–[26] have demonstrated that IL-10 and the JAK / STAT signaling pathway play important roles in DCs maturation.

Previous studies have suggested that several soluble factors, such as IL-6 [11], IDO [10], [27], PGE2 [6], [10], and NO [28], are involved in this process. However, the mechanism(s) by which MSCs exert their inhibitory effects on the maturation of DCs is still poorly understood. In the following experiments, we cultured MSCs and DCs within different culture media and under various conditions. Then, we established co-cultures of the two cell types using Transwell plates. In some experiments, we added IL-10, IL-10NA and AG490 to the co-culture medium to probe the role of the IL-10 and JAK1/STAT3 signaling pathways in the inhibitory mechanisms of MSCs on DCs. FACS, ELISA and Western blotting were used to characterize the cell cycle, cytokine production and protein expression, respectively. Based on our findings, we propose an IL-10 feedback loop is involved in the inhibitory effect of MSCs on DCs. In the co-culture, IL-10 secretion increased significantly, compared with MSCs or DCs alone. Furthermore, co-cultures activated the JAK1 / STAT3 signaling pathway, inhibiting the maturation of DCs, and affecting IL-12 secretion from DCs. Moreover, we report for the first time that IL-10 and the JAK1 / STAT3 pathway play important roles in MSCs-mediated inhibition of DCs maturation.

## Methods

### Animals

Male Sprague Dawley (SD) rats weighing 60–80 g were cared for in accordance with US National Institutes of Health published guidelines published by the National Institutes of Health. All of the study procedures were approved by the Harbin Medical University Institutional Animal Care and Use Committee. The study was conducted in compliance with the Guide for the Care and Use of Laboratory Animals published by the National Academy Press (NIH, revised in 1996).

### Isolation, Culture and Characterization of MSCs

The MSCs were isolated and cultured from the rat bone marrow of the femur and tibia [6]. Bone marrow cells were plated in culture flasks at a concentration of 10^6^ cells/mL in DMEM/F-12 (1∶1) (Hyclone, Logan, UT), supplemented with 10% fetal calf serum (FCS; Hyclone) and 1% penicillin/streptomycin, at 3×10^5^/cm^2^ at 37°C in 5% CO_2_ humidified atmosphere. At 80–90% confluence, MSCs were treated with trypsin and further expanded at a ratio of 1∶2. MSCs were used in the experiments only after 3–5 expansion passages, to ensure depletion of monocytes/macrophages. MSCs were characterized by flow cytometric analysis for the expression of the typical markers, CD29, CD90, and CD44, and the absence of the hematopoietic markers CD45 and CD34. All data are expressed as percentages from FACS measurements.

### Culture, Generation and Characterization of DCs

We cultured DCs in accordance with our protocol previously described in detail elsewhere [29]. Like the MSCs, DCs were also derived from the rat femur and tibia bone marrow. In the course of the isolation, we added 5 mL red blood cell lysate (Beyotime, China) to the cell suspension. After cleavage at room temperature for 5 min, the cell mixture was centrifuged (1000 rpm, 5 min). Cells were then cultured in 6-well plates using RPMI 1640 medium supplemented with 10% FCS, 1% penicillin/streptomycin, recombinant rat GM-CSF (50 ng/mL), and IL-4 (50 ng/mL) (PeproTech, Rocky Hill, NJ). After 5 days, cultured cells were harvested by gentle aspiration and analyzed by flow cytometry to assess the immature DCs (iDCs) phenotype. DCs maturation was induced by stimulation with lipopolysaccharide (LPS, Sigma). After LPS (200 ng/mL) stimulation for 48 h, DCs were analyzed by flow cytometry for CD80, CD86, OX62, MHC-II and CD11b/c to assess whether the mature phenotype (mDCs) was successfully induced.

### Transwell Co-cultures of MSC-DC

A Transwell system (0.8-µm pore size membrane, Corning, Acton, MA) was used to prevent MSCs from contacting directly the DCs. MSCs and iDCs were placed in the upper and lower layers of the Transwell plate, respectively, at various ratios (1∶1, 1∶10, and 1∶100). Each well in a 6-well Transwell co-culture plate contained 5×10^5 ^DCs in RPMI 1640 medium, supplemented with 10% FCS, 1% penicillin / streptomycin, recombinant rat GM-CSF (50 ng/mL), and IL-4 (50 ng/mL). LPS (200 ng/mL) was added to the DCs layer for 2 additional days (48 h) to stimulate iDCs maturation in the presence or absence of MSCs. In some experiments, IL-10 (500 ng/ml; PeproTech) was added to the MSC layer for 48 h. To investigate whether MSCs exerted their inhibitory effect on DCs differentiation by IL-10 production, IL-10NA (5 µg/mL; Abcam, Cambridge, UK) was added to the co-cultures for 48 h. To distinguish the exogenous IL-10 added to the culture from the endogenous IL-10 produced by the cells, IL-10 (500 ng/ml) and LPS (200 ng/mL) was added to iDCs monoculture, or IL-10NA (5 µg/mL) followed by IL-10 was added to iDCs-LPS. In another group, AG490 (40 µmol/L; Beyotime, China) was added to the co-culture for 48 h to investigate the role of the JAK1 / STAT3 signaling pathway in the effects of MSCs on DCs.

### FACS

For the analysis of the cell surface-marker expression, cells were digested by trypsin, washed twice with phosphate-buffered saline (PBS), and kept at 4°C in the dark until analysis. For MSCs, the following rat antibodies (Abs) were used: Phycoerythrin-cy5 (PE-cy5)-labeled anti-CD45, PE-anti-CD90, Fluorescein Isothiocyanate (FITC)-labeled anti-CD44, anti-CD29 (BD Pharmingen, USA) and Alexa Flour 647-labeled anti-CD34 (eBioscience, San Diego, CA). Like the MSCs, DCs were harvested by incubation in ice-cold PBS for 30 min. Cells were stained with antibodies against CD80, OX62 and CD11b/c (PE-labeled), and CD86 and MHC-II (FITC-labeled; eBioscience). As a control, cells were stained with mouse IgG1 isotype-control antibodies. DCs were combined with MSCs in various ratios, and we measured changes in CD80, OX62, CD86, MHC-II and CD11b/c. Cells were analyzed using a FACScan (BD Biosciences, Franklin Lakes, NJ, USA) with the CellQuest Analysis (BD Biosciences) and FlowJo software (TreeStar). Results are expressed by the percentage of positively stained cells relative to total cell number.

### ELISA

The supernatants of MSCs and DCs cultures, and also of the co-cultures were collected respectively in 1.5 ml micro-tubes and kept at −20°C. IL-10 quantification was performed in the supernatants of the co-cultures at 48 h. To measure IL-12 production by mDCs, culture supernatants were collected at day 7 (5 d + 48 h after the LPS stimulation). The measurement was conducted according to the manufacturer’s protocol. Detection limits were 7.8 pg/mL for IL-12 and 7.7 pg/mL for IL-10. All determinations were made in triplicates. IL-10 and IL-12 ELISA kits were purchased from the Xitang Company (Shanghai, China). ELISA plates were read at OD450 on a Microplate ELISA reader (Autobio Diagnostics Co. Ltd, China).

### Immunofluorescence

To investigate the secretion of IL-10 from MSCs and DCs in Transwell co-culture plates, we designed a cell immunofluorescence study of monocultures of MSCs and of mDCs, and co-cultures of MSCs and iDCs (1∶10) plus LPS. Both cell types were grown on glass coverslips and fixed with 4% paraformaldehyde for 30 min at room temperature, permeabilized with 0.3% Trition-X100, blocked with goat serum and incubated with anti-IL-10 antibody (1∶200, ab9969, Abcam) overnight at 4°C. After washing, the cells were incubated with the Alexa Fluor 555 goat anti-rabbit IgG (1∶500, Invitrogen Technology, USA) for 2 h at 37°C. The nuclei of cells were counterstained with 4′,6-diamidino-2-phenylindole (DAPI) (0.1 µg/ml, Sigma). The fluorescence images were acquired with a confocal laser-scanning microscope (Olympus FluoView V5.0 FV1000).

### Western Blotting

DCs were washed with ice-cold PBS. After at least 30 min on ice, insoluble components were removed by centrifugation (12,000 rpm, 4°C, 15 min). Proteins were separated by 10% sodium dodecyl sulfate–polyacrylamide gel electrophoresis (SDS-PAGE), and transferred onto nitrocellulose membranes. Total protein concentration was measured using the bicinchoninic acid assay, with bovine serum albumin (BSA) used to construct the standard curve. Nonspecific binding was blocked by incubating the membranes with 5% nonfat dry milk and TBST (0.05% Tween 20 in Tris-buffered saline, TBS). Membranes were incubated overnight at 4°C with anti-JAK1 mAb ( monoclonal antibody,3344,Cell Signaling Technology, Danvers, MA, USA), anti-STAT3 (9132, Cell Signaling Technology), anti-phospho-JAK1 mAb (ab5493, Abcam), or anti-phosphor STAT3 mAb (Tyr705, Cell Signaling Technology) at an appropriate dilution(1∶1000 in each Ab). Subsequently, the membranes were washed in TBST and incubated with horseradish peroxidase-conjugated secondary antibodies for 1 h at room temperature. Specific protein bands were visualized on film by enhanced chemiluminescence (ECL) (Applygen Technologies Inc., China) following the protocol of the manufacturer. The bands were quantified by scanning densitometry using a GS-710 Imaging Densitometer (Bio-Rad, Hercules, CA) and normalized to that of β-actin. All data was obtained in triplicate independent experiments.

### Statistical Analysis

Descriptive and analytical statistics were performed using SPSS software (ver. 15; Chicago, IL). Values for all measurements are presented as mean ± standard deviation (SD). Comparisons for two pairs were performed using the Student’s *t*-test. Values of *p*< 0.05 were considered to indicate statistically significant differences.

## Results

### MSCs Assessed by Morphology and FACS

The plastic-adherent cells under standard culture conditions obtained from rat bone marrow (MSCs) showed the typical spindle-shape. The MSCs were expanded for 3–5 passages in a plastic dish, and exhibited a typical fibroblastic morphology. The percentage of the MSCs obtained from culturing bone marrow cells was 99.04%. MSCs at passage 5 were analyzed for the expression of cell surface molecules by flow cytometry. As reported in other studies [3], [4], MSCs express CD29 and CD90, partly express CD44, but show negative expression of CD34 and CD45. We detected the expression of CD29 (99.04%), CD90 (88.27%), CD44 (35.65%), CD34 (0.84%), and CD45 (2.13%) in MSCs, respectively (Fig. 1). Thus, these cells have the typical expression profile of MSCs.

**Figure 1:** Cell surface markers of MSCs. The surface marker molecules expressed by the Passage 5 culture of MSCs were analyzed by flow cytometry. (B) Quantification by image analysis of the positive cells. The numbers in the histograms indicate the mean fluorescence of each MSC markers. (C) Percent of MSCs obtained from culturing bone marrow cells.

### MSCs Inhibition of DCs Maturation Stimulated by LPS

Myeloid cells purified from Sprague Dawley rat bone marrow were cultured in medium with GM-CSF and IL-4 to induce DCs differentiation. After 5 days, DCs differentiation was assessed by analyzing the expression of OX62, MHC-II, CD11b/c and of the co-stimulatory molecules, CD80 and CD86. iDCs at 5 days were positive for CD80 (64.02%), CD86 (69.55%), OX62 (86.62%), MHC-II (61.05%) and CD11b/c (60.50 %), (Fig. 2A). These iDCs were stimulated by LPS for 48 h to acquire the mature phenotype (mDCs). mDCs showed significantly increased expression levels of the same panel of markers CD80 (91.38%), CD86 (88.04%), OX62 (93.33%), MHC-II (91.06%) and CD11b/c (79.84%) (Fig. 2B). However, when mDCs are co-cultured with MSCs, and stimulated with LPS, the cells displayed a phenotype similar to those of iDCs. For example, at a ratio of MSC: DC of 1∶10, the expression of CD80, CD86, OX62, MHC-II and CD11b/c was 65.46%, 55.05%, 70.19%, 66.63%, and 66.64%, respectively (Fig. 2C). A maximal inhibitory effect could be observed at a 1∶1 DC: MSC ratio. The inhibitory action was decreased at a 100∶1 ratio. Thus, the effect of MSCs on the maturation of DCs features a dose-dependent relationship.

**Figure 2:** Phenotype analysis of different DCs. (A) FACS histograms showed the expression of cell surface markers on iDCs, which expressed low levels of CD80, MHCII, OX62, CD86 and CD11b/c. OX62 expressed much higher than other makers, because OX62 is an important marker of rat DCs. (B) LPS- stimulated mature DCs (mDCs) showed about equally up-regulated levels of all markers. Except CD86, three makers showed above 90 percent expression. (C) MSC-DC-LPS-activated DCs in co-culture expressed lower levels of the four markers compared with mDCs, but the expression was slightly higher when compared with iDCs. This result suggests that MSCs inhibit DCs phenotype expression (MSC:DC = 1∶10). Data represent mean fluorescence intensity for the surface density of markers. (D) Quantification by image analysis of the positive cells. The numbers in the histograms indicate the mean fluorescence of each DCs markers. *P<0.05(mDC group versus iDC group), #P<0.05(MSC-DC group versus mDC group).

### MSCs Inhibition of IL-12 Secretion by DCs in Co-culture

iDCs were cultured in the presence and absence of MSCs after 48 h, and mDCs supernatants were collected for cytokine quantification. Using ELISA, we analyzed the amount of IL-12 secreted by these cells. As shown in Figure 3A, MSCs produced a small amount of IL-12 (13.67±4.34 pg/mL). iDCs secreted significantly more IL-12 (56.07±14.83 pg/mL) compared with MSCs alone. Larger amounts of IL-12 (413.3±93.99 pg/mL) were released by mDCs cultured alone (P < 0.05; Fig. 3A), while much lower amounts were produced by DCs co-cultured with MSCs (72.1±21.41 pg/mL), which are comparable to levels of IL-12 secreted by iDCs in monoculture.

**Figure 3:** IL-10 and IL-12 secretion as assessed by ELISA. (A) IL-12 secreted in monocultures of MSCs, iDCs and mDCs and in the co-culture of MSC-DC (MSC:DC = 1∶10). (B) IL-10 secreted in monocultures of MSCs, iDCs and mDCs and in the co-culture of MSC-DC (MSC:DC = 1∶10). *P<0.05(mDC group versus iDC group), #P<0.05(MSC-DC group versus MSCs group).

### MSCs Secretion of IL-10 in Co-culture

Co-culture supernatants were collected for analysis of IL-10 expression via ELISA. The supernatants of MSCs cultured alone were associated with a small amount of IL-10 (8.57±1.26 pg/mL). The DCs in monoculture, both iDCs and mDCs, also secreted low amounts of IL-10 (16.53±3.25 and 54.77±12.42 pg/mL, respectively). However, the IL-10 expression level in MSCs was increased significantly (583.37±100.81 pg/mL) when DCs were present in the co-culture (in a ratio of 1∶10) (Fig. 3B).

### Immunofluorescence Assay

The expression of IL-10 was very weak in the monoculture of MSCs. The monoculture of DCs showed higher expression of IL-10 than the monoculture of MSCs. In the co-culture of MSCs and DCs (ratio 1∶10), the MSCs showed a clear increase in IL-10 expression when compared with the monoculture. When compared with DCs in monoculture, the DCs in co-culture plate do not overexpress IL-10 significantly. It is clear that in the co-culture condition the MSCs expressed significantly more IL-10 than DCs (Fig. 4 A, B, C, D).

**Figure 4:** Immunofluorescence staining of MSCs, DCs and both cells in co-culture plates with IL-10. (A) Monoculture of MSCs. (B) MSCs in Transwell co-culture with DCs. (C) Monoculture of iDCs-LPS. (D) iDCs-LPS in Transwell co-culture with MSCs (MSC:DC = 1∶10). Red staining shows IL-10 expression; DAPI blue staining of cell nuclei. Scale bar 251658240 = 251658240100 µm.

### DCs Expression of (Phospho-) JAK1 and (Phospho-) STAT3 in the Presence of MSCs

We collected DCs, iDCs, mDCs, and DCs co-cultured with MSCs. From all of these cells, the protein was extracted and analyzed using Western Blotting to detect the expression of JAK1, STAT3, phospho-JAK1, and STAT3 (P-JAK1 and P-STAT3). We found that MSCs could enhance the expression of JAK1, STAT3, phospho-JAK1, and STAT3 in DCs (eg.P-JAK1 2.367 in the MSC-DC group, 1.125 and 1.253 in iDCs and mDCs, respectively, p<0.05; Fig. 5 A, B).

**Figure 5:** Protein expression of JAK1, P-JAK1, STAT3 and P-STAT3 in monocultures of iDCs, mDCs and in co-cultures of MSC-DC (MSC:DC ratio of 1∶10). (A) Western Blot; (B) Quantification by image analysis of the protein expression. * P<0.05 (MSC-DC group versus mDC group).

### IL-10 and IL-12 Secretion in the Presence of IL-10, IL-10NA and AG490

To examine the effect of IL-10 and JAK1/STAT3 signaling pathways on DCs activity, we added IL-10, IL-10NA and AG490 to the MSCs layer in co-culture plates for 48 h, respectively. Cell supernatants were collected and analyzed by ELISA to characterize the secretion of IL-10 and IL-12. The results showed that IL-10 levels in the IL-10 group (630.97±110.38 pg/mL) increased even more than in the MSC-DC co-culture group (583.37±100.81 pg/mL). IL-10NA added into the co-culture system successfully reduced the IL-10 level (126.4±29 pg/mL). In the presence of AG490, a JAK inhibitor, the level of IL-10 secretion also decreased, to a degree that was similar to the effect of IL-10NA. (Fig. 6A). IL-12 levels decreased in the IL-10 (64.43±15.59 pg/mL) and in the IL-10NA group (98.83±32 pg/mL) by comparison to mDCs (413.3±93.99 pg/mL, Fig. 3A). When AG490 was added to the system, IL-12 levels (149.7±78.42 pg/mL) increased compared to that in IL-10 group, but still remained much lower than levels of IL-12 released from mDCs (Fig. 6B). In DC-IL-10 group, IL-10 and IL-12 secreted 548.22± 86.45 and 68.49±10.64 pg/mL, respectively, while in DC -IL-10-IL-10NA group data were 78.86±23.09 and 377.38±102.29 pg/mL, respectively (Fig. 6A, B).

**Figure 6:** ELISA analysis of co-cultures of MSC-DC supplementated with exogenous IL-10, IL-10NA and JAK inhibitor (AG490). IL-10 and IL-12 levels in DC–IL-10 and DCs -IL-10 -IL-10NA group by ELISA. (A) IL-12; (B) IL-10.* P<0.05 (IL-10NA group versus MSC-DC group), # P<0.05 (AG490 group versus MSC-DC group), & P<0.05 (DC- IL-10 group versus MSC-DC group), § P<0.05 (DC- IL-10-IL-10NA group versus IL-10NA group),$ P<0.05 (DC- IL-10-IL-10NA group versus DC- IL-10 group).

### Phenotype of DCs in the Presence of Exogenous IL-10, IL-10NA and AG490

To investigate the mechanism(s) involved in the MSC-mediated inhibition of DC differentiation, we added IL-10, IL-10NA and AG490 to the co-cultures. Using this approach allowed us to elucidate whether IL-10 and/or the JAK1/STAT3 signaling pathways play a role in this mechanism. As shown in figure 6, CD80, CD86, OX62, MHC-II and CD11b/c showed reduced expression in the IL-10 group. When IL-10NA was added to the co-culture medium, as expected, IL-10NA strengthened the expression of these markers. AG490 reduced CD80, CD86, OX62, MHC-II and CD11b/c expression levels compared with the MSC-DC co-culture (Fig. 7A, B, C, F).

**Figure 7:** DCs surface markers (CD80, CD86, OX62, MHC-II and CD11b/c) in the MSC-DC co-culture system (ratio MSC:DC of 1∶10) supplemented with exogenous: (A) IL-10; (B) IL-10NA and (C) AG490. (D, E) These makers expression in DC-IL-10 and DC - IL-10 - IL-10NA group by FACS. (F, G) Quantification by image analysis of the positive cells. Numbers in the histograms indicate the mean fluorescence of each DCs markers. *P<0.05(IL-10 group versus MSC-DC group), # P<0.05(IL-10NA group versus MSC-DC group), $ P<0.05(AG490 group versus MSC-DC group).

In DC-IL-10 group, the expression of CD80, CD86, OX62, MHC-II and CD11b/c was 69.62%, 62.56%, 76.03%, 57.16%, and 57.99%, respectively. However, in DC-IL-10 -IL-10NA group, the makers of CD80 (88.11%), CD86 (65.65%), OX62 (81.94%), MHC-II (78.75%) and CD11b/c (72.97%) expressed higher than in DC-IL-10 group (Fig. 7 D, E, G).

### Expression of (Phospho-) JAK1 / STAT3 in the Presence of IL-10, IL-10NA and AG490

We aimed to test the hypothesis that the IL-10 and JAK1/STAT3 pathway have a major role in MSC-mediated inhibition of DCs maturation. To address this hypothesis we studied the effect of exogenous IL-10, IL-10NA and AG490 on the expression of (phospho-) JAK1 / STAT3 in co-cultures of MSC-DC. Surprisingly, we observed that by adding IL-10 to the co-culture, the expression of total JAK1/STAT3 and phospho-JAK1 / STAT3 was enhanced. (Fig. 8A, B). As expected, in the presence of IL-10NA, the expression of all these markers (total JAK1/STAT3 and phospho-JAK1/STAT3) was reduced. In the DC-IL-10 group, total JAK1/STAT3 and phospho-JAK1/STAT3 were overexpressed when compared with the monoculture of DCs, but showed weaker expression than those of MSC-DC-IL-10 in the co-culture. When IL-10NA was added to the DC-IL-10 plates, the expression of those antibodies showed a decrease. (Fig. 8 C, D) Similar to the effect of IL-10NA, AG490 also reduced the expression of total JAK1/STAT3 and phospho-JAK1/STAT3 (Fig. 8 E, F). The expression levels of phospho-JAK1/STAT3 are significantly weaker than total JAK1/STAT3.

**Figure 8:** Protein expression of JAK1, P-JAK1, STAT3 and P-STAT3 of DCs in co-cultures of MSC-DC (MSC:DC ratio of 1∶10). (A) Western Blotting of the co-culture, without supplementation, or supplemented with, IL-10 or with IL-10NA (P<0.01); (B) Quantification by image analysis of the protein expression in the same conditions as (A); (C) Western Blotting of the co-culture, without supplementation, or supplemented withAG490 (P<0.01); (D) Quantification by image analysis of the protein expression in the same conditions as in (C). (E) Western Blotting of DC -IL-10 and DC- IL-10 -IL-10NA (P<0.01); (F) Quantification by image analysis of the protein expression in the same conditions as in (E). * P<0.05(IL-10 group versus MSC-DC group), # P<0.05(IL-10NA group versus MSC-DC group), $ P<0.05 (AG490 group versus MSC-DC group), & P<0.05 (DC- IL-10 group versus DC group), § P<0.05 (DCs- IL-10-IL-10NA group versus DC group).

## Discussion

MSCs have been shown to potently suppress immunological activity by acting on various cells of the immune system. Additionally, many reports have documented a potent inhibitory effect of MSCs on myeloid or monocyte DCs maturation [6]–[7]. These inhibitory mechanisms involve two aspects: cell-to-cell contact, and secretion of specific cytokines. Several studies have previously demonstrated that the expression of IL-10 is significantly increased when MSCs and T cells are co-cultured in a Transwell system. Thus, we hypothesized that MSCs may inhibit DCs maturation through the action of the cytokine IL-10. It is well known that IL-10 is a suppressive cytokine being implicated in the proliferation and on the cytokine production of T cells. IL-10 has also been shown to have a role in inducing T cell anergy (a tolerance mechanism in which the lymphocyte is intrinsically functionally inactivated, in a hyporesponsive state) [22]. Thus, IL-10 may also inhibit DCs maturation and function. However, in MSC-DC co-cultures, and in the presence of IL-10, we observed that the expression of cytokines is increased markedly. In addition, we provide evidence by cell immunofluorescence that the MSCs secreted more IL-10 than the DCs in the Transwell co-cultures (Figure 4). This result shows that the mechanisms underlying the MSCs and the IL-10 inhibitory effect are still poorly understood, being necessary to study them in greater detail.

In the current study, we cultured and characterized MSCs and DCs in monoculture, and in co-cultures using Transwell plates. We aimed to use this culturing platform (DCs and MSCs co-cultured in the Transwell two-chamber system) to exclude the effect of cell-to-cell contact from our experiments. Under these culture conditions, a significant inhibition of DCs differentiation was observed at day 5 or 7, suggesting that soluble factors may be involved in this inhibitory mechanism. We found that there was a robust increase in the expression of IL-10 in the supernatants of co-cultures (583.37±100.81 pg/mL) compared with monocultures of MSCs (8.57±1.26 pg/mL) or DCs (either iDC: 16.53±3.25 pg/mL or mDC: 54.77±12.42 pg/mL).

The JAK-STAT signaling pathway was also analyzed in detail to evaluate the mechanism of action of IL-10. Using Western blotting, our results showed that JAK1, P-JAK1, STAT3, and P-STAT3 were all overexpressed when either MSCs or IL-10 was added to the co-culture medium. The expression levels are also much higher than those observed in monocultures of DCs (iDCs or mDCs). Additionally, we noticed that the MSCs group (MSC:DC = 1∶10) had greater cytokine expression than other groups using different proportions of the two cell types (1∶1 or 1∶100). The MSCs, particularly at the highest ratio in the co-culture (1∶10), could reproduce the inhibition patterns without cell-cell contact in the Transwell system. In the IL-10 group, the expression of JAK1 and STAT3 was higher compared with the MSCs group. A possible reason for this effect is that IL-10, when associated with MSCs [30] in the co-culture system, may enhance the expression of JAK1 and STAT3, which synergistically contribute to inhibition of DCs maturation.

The MSC-mediated inhibition of DCs maturation may also affect the expression of DCs surface markers, and on the development of DCs function, such as IL-12 production. Our data suggests that MSCs can suppress the secretion of IL-12 by DCs. Additionally, we analyzed the expression of CD80, CD86, OX62, MHC-II, and CD11b/c as these are considered to be markers of DCs maturation. We observed that the expression of these markers declined in the presence of MSCs. This result suggests that the presence of MSCs in co-culture directly interferes with the maturation of DCs.

We analyzed the involvement of IL-10 on the inhibitory effect of MSCs on the maturation of DCs. To assess this effect, IL-10 or IL-10 neutralizing antibody were added into the DCs monoculture or MSC-DC co-cultures in the Transwell system. ELISA results show that IL-10 was overexpressed in the IL-10 supplemented group, and markedly decreased in the IL-10NA group, as expected. We also observed that the expression of CD80, CD86, OX62, MHC-II and CD11b/c (panel of positive markers for DCs maturation) declined in the IL-10 group, while the expression of those markers was restored to baseline levels in the IL-10NA group. This result confirms that in the presence of MSCs, or in the presence of IL-10, a similar inhibitory pattern is observed. Exogenous IL-10 and the presence of MSCs seem to have a synergistic effect. Furthermore, the presence of IL-10NA in the co-culture reverses the inhibition.

Based in our results, we propose the concept of an IL-10 feedback loop mechanism of control for the maturation of DCs (Fig. 9). This feedback loop, helps in explaining the mechanism of increase of IL-10 expression that we have reported. MSCs or DCs in monoculture secrete low amounts of IL-10. When these cells are in co-culture, IL-10 combines with the IL-10 receptor and further activates the JAK-STAT signal transduction pathway [26]. Once activated (by LPS), this signaling pathway led to decreased IL-12 secretion. Simultaneously, DCs maturation was inhibited; the number of iDCs increased, and conversely the number of mDCs decrease. That is, the pool of immature DCs is enlarged at the expense of mature DCs. Our data suggest that mDCs can secrete more IL-10 than iDCs, which is consistent with previous results reported in the literature [18]. Thus, in the supernatants of co-cultures, fewer iDCs secrete lower amounts of IL-10. Moreover, more IL-10 may be produced through a positive loop. Accordingly, we observed a marked increase on the levels of IL-10 in MSC-DC co-culture medium supernatants.

**Figure 9:** Newly proposed IL-10 feedback loop. The figure illustrates the interplay between IL-10 and the JAK1/STAT3 signaling pathway involved in mechanism inhibition of DCs maturation by MSCs. The MSCs facilitate the combination of the cytokine IL-10 with its IL-10 receptor. This complex activates the JAK1/STAT3 signaling pathway that suppresses the DCs maturation. This inhibition of maturation causes a decrease in the expression of IL-10. Thus, the levels of the cytokine IL-10 command this positive feedback loop.

Our results showed that MSCs, IL-10, JAK-STAT, and DCs are all connected to each other. In previous reports, differing soluble factors (PGE_2_, IDO, IL-6 [6], [10], [11], [27]) and signaling pathways (Notch [31], toll-like receptor (TLR) [32]) have been suggested to mediate the inhibitory effect exerted by MSCs on the activity of DCs. However, to the best of our knowledge, this is the first report establishing a link between the levels of the cytokine IL-10, and the JAK-STAT signaling pathway with respect to the mechanism of inhibition of MSCs on DCs. We postulate that the MSCs specifically inhibit DCs function and maturation through IL-10 and the JAK-STAT signaling pathway.

In this study, we investigated the JAK-STAT signaling pathway with regard to the inhibitory mechanism of action of MSCs on the maturation of DCs. Our study did not focus on effects at the protein level, for example, the implication of the suppressor of cytokine signaling (SOCS) [33]. Additionally, this study was only performed *in vitro*. Our data needs to be confirmed by *in vivo* data. To date, our studies only discuss IL-10 and JAK-STAT, without involvement of other cytokines or signal transduction pathways. It is possible that other cytokines and signaling pathways may also be implicated in the inhibitory mechanism of action of MSCs on DCs.

In summary, our present study provides novel information on the molecular mechanisms and on the timing of MSCs-mediated inhibition of DCs maturation and function. Our data suggests that MSCs may modulate the immune system, not only through acting directly on T cells, but also in the first step of the immune response through the inhibition of DCs differentiation and maturation. We report data supporting the existence of a link between the cytokine IL-10 and the JAK-STAT pathway. This inhibition may have interesting implications, for example in the transplantation of MSCs to inhibit the maturation of DCs and reduce the incidence and degree of severity of graft-versus-host disease (GVHD). This study may open new, clinically-relevant, research avenues. A pioneering clinical study by Le Blanc *et al* [34] revealed that the infusion of MSCs could successfully treat severe acute GVHD. Because DCs play a central role in the induction of T cell-mediated transplant rejection or GVHD [35], we studied the inhibitory mechanism of MSCs activity on DCs. These findings may enhance the future prospects of the clinical application of MSCs in new and broader immune-related applications. An understanding of the mechanism(s) of action may allow the translation of basic knowledge of MSCs biology into the design of new clinical therapies. Ongoing and future clinical trials with MSCs will provide a rich source of bedside information that can be extended in the laboratory to further advance this important field of research.
